# A Three-mRNA Signature Associated with Pyrimidine Metabolism for Prognosis of BRCA

**DOI:** 10.1155/2022/7201963

**Published:** 2022-02-16

**Authors:** Xiaoxue Zhang, Qiang Zhang, Xianxin Xie, Yang Li, Zhiyuan Pang, Tao Yu

**Affiliations:** ^1^Department of Medical Imaging, Cancer Hospital of China Medical University, Liaoning Cancer Hospital & Institute, No. 44 Xiaoheyan Road, Dadong District, Shenyang, 110042 Liaoning Province, China; ^2^The Second Department of Breast Surgery, Cancer Hospital of China Medical University, Liaoning Cancer Hospital & Institute, Shenyang, Liaoning Province, China; ^3^Department of Breast Surgery, Cancer Hospital of China Medical University, Liaoning Cancer Hospital & Institute, Shenyang, Liaoning Province, China

## Abstract

**Objective:**

Breast invasive carcinoma (BRCA), as a systemic disease, is currently the most malignant tumor among women. Early detection of BRCA will increase the probability of cure. Pyrimidine metabolism (PyM) stands for an essential metabolic pathway related to DNA replication of cancer cells, which may also serve as a diagnostic marker and therapeutic target. Therefore, the aim of this research is to discover a prognostic signature associated with PyM for BRCA.

**Methods:**

The BRCA mRNA sequencing data along with microarray data were obtained based on The Cancer Genome Atlas (TCGA) database. In addition, 4 PyM-related gene sets were profiled through gene set enrichment analysis (GSEA); it revealed the core genes differentially expressed in cancer and paracancerous tissue. Thereafter, genes were subjected to univariate as well as multivariate regression for constructing an mRNA signature to independently predict BRCA prognosis. Then, the Kaplan-Meier (KM) curve was applied for validation. The prognostic power of the signature was verified against the METABRIC (Molecular Taxonomy of Breast Cancer International Consortium) database.

**Results:**

We constructed a three-mRNA (RRM2B, NME3, and POLD2) gene signature related to PyM to predict overall survival (OS) for BRCA. The as-constructed gene signature was adopted to classify cases as high- or low-risk group, identifying patients with BRCA with poor prognosis. Additionally, the risk score obtained using our constructed 3-mRNA prognosis signature is independent from other clinical variables.

**Conclusion:**

Our findings suggested that PyM-related mRNA signature might be a combined prognostic biomarker for BRCA and can provide important reference that are useful for individualized treatment for BRCA patients.

## 1. Introduction

Nucleotide metabolism is a critical pathway that generates purine and pyrimidine molecules for DNA replication, RNA synthesis, and cellular bioenergetics [1]. The increasing metabolism of nucleotides facilitates out-of-control tumor growth, which serves as a cancer hallmark [2]. There has been an explosion of knowledge in disorders of pyrimidine metabolism during the last 20 years [3]. Pyrimidines have long been considered building blocks in synthesizing nucleic acids as well as intermediates for metabolic energy transfer. Growing attention has been paid to pyrimidines since their genetic alterations in metabolism are associated with different symptoms (like immunodeficiency, hyperuricemia, and even neurological disorders) [4]. PyM represents a complicated enzyme network, which combines salvage and de novo synthesis of nucleotides, along with catalytic pyrimidine degradation [5]. PyM contains 3 related pathways shown below: (1) free base and nucleoside salvage, (2) de novo synthesis based on ribose precursors and amino acids, and (3) excessive nucleoside and nucleotide catabolism [6]. Early success in cancer metabolism took advantage of this characteristic by making cancer cells vulnerable to inhibition of this pathway [7]. The importance of intact pyrimidine pathways in human physiology and their upregulation in malignancy [8] makes them ideal targets for pharmacological interventions. Agents inhibiting the synthesis and incorporation of nucleotides in DNA are widely used as chemotherapeutics to reduce tumor growth, cause DNA damage, and induce cell death [9]. Heidelberger and colleagues designed fluorinated uracil-based pyrimidine analogues, which disrupted tumor DNA biosynthesis and which are to this day used to treat colorectal and breast cancer [10, 11].

BRCA is a malignant tumor in which cancer cells have penetrated the basement membrane of the breast ducts or lobular acinars and invaded the interstitium. The vast majority of breast invasive carcinoma is adenocarcinomas, which originate from the parenchymal epithelial cells of the breast, especially the peripheral ductal lobular units of the breast [12]. Ninety-nine percent of BRCA patients are women, so this disease is the malignant tumor with the highest incidence among women [13]. Among the known risk factors for BRCA, in addition to age factors, individual family history, menstrual history, pregnancy history, and benign breast lesions are all closely related to the risk of breast cancer [14]. Early detection and early diagnosis of this disease is the key to improving the efficacy and can significantly extend the survival period [15]. Clinically, there is always a need for better or alternative methods to identify people at risk of cancer [16]. Previous studies have found many prognostic biomarkers in patients with BRCA [17]. However, there is little research on the systematic study of metabolic status as well as prognostic significance among tumor cases, in particular for research associated with PyM, and this is possibly a novel point cut in our study. Therefore, in this study, we are trying to exploit the gene signature associated with PyM in BRCA.

This work carried out GSEA for identifying the gene sets associated with PyM to differentiate clinical as well as molecular parameters for BRCA. We developed a PyM-related prognostic signature (RRM2B, NME3, and POLD2) with whole genome expression data from TCGA database. Surprisingly, the local PyM-related risk signature could independently classify patients with BRCA with a high risk of unfavorable outcome. Then, the prognostic power of the signature was validated in the METABRIC database. Our finding provides important references to understand the mechanism of PyM and to develop an individualized treatment for BRCA patients.

## 2. Materials and Methods

### 2.1. Collection of Gene Expression Data and Patient Clinicopathological Parameters

The whole mRNA expression data and corresponding clinical parameters of BRCA were extracted from TCGA (http://cancergenome.nih.gov/) and METABRIC database. METABRIC is a Canada-UK joint project that is aimed at further classifying breast tumors based on molecular characteristics that help determine the best course of treatment. Altogether, 1108 BRCA cases together with 113 normal subjects who had matched clinical characteristics were obtained from TCGA.  Table 1 shows the clinical characteristics of all participants. And we collected 1892 BRCA samples from the METABRIC database.

### 2.2. Functional and Pathway Enrichment Analysis

GSEA (http://www.broadinstitute.org/gsea/index.jsp) can be applied to examine the significance of gene set-derived genomes in two gene expression data groups [18]. We discovered three PyM-related gene sets on the GSEA website, which were called GO_PYRIMIDINE_CONTAINING_COMPOUND_CATABOLIC_PROCESS, GO_PYRIMIDINE_CONTAINING_COMPOUND_BIOSYNTHETIC_PROCESS, KEGG_PYRIMIDINE_METABOLISM, and GO_PYRIDINE_CONTAINING_COMPOUND_METABOLIC_PROCESS in Molecular Signatures Database v4.0 (http://www.broadinstitute.org/gsea/msigdb/index.jsp). Gene sets were determined by the corrected *p* value (*p* < 0.05) in subsequent analysis. Thereafter, we also screened core genes (core enrichment: yes) in subsequent analysis. Later, the above screened genes were subjected to functional enrichment analysis by the bioinformatics approach Metascape (http://metascape.org). The aim of Metascape is to develop a set of reliable, productive, and intuitive tools that help the biomedical research communities to analyze gene/protein lists and make better data-driven decisions [19].

### 2.3. Establishment and Confirmation of a Prognostic Signature

Figure 1 displays the flowchart of the present work. In this study, we used the univariate Cox model to calculate the association of every screened PyM-related mRNA expression with patient OS. After that, the multivariate Cox analysis method was used to evaluate the weight of mRNA, and the prognostic gene from the previous step was further analyzed and confirmed as a factor to independently predict prognosis. Afterwards, we determined the risk scores for all BRCA cases according to mRNA expression as well as the regression coefficients acquired upon multivariate Cox regression. Risk score = gene 1 expression level × *β*1 + gene 2 expression level × *β*2 + ⋯+gene *n* expression level × *βn*. In addition, R package was utilized for exploring the relationship between risk scores and OS. Thereafter, the median risk score value was adopted as the threshold for classifying 1108 BRCA cases as a high- or low-risk subgroups. KM curves were used for survival analysis of single genes.

### 2.4. Statistical Analysis

GraphPad Prism 7 and SPSS 16.0 were utilized for statistical analysis. At the same time, for prognostic genes in BRCA, their genetic alterations were determined using the cBioPortal web software (http://www.cbioportal.org/). The chi-square test was used to demonstrate the relationship between risk score and clinical parameters.

## 3. Results

### 3.1. Genes from the PyM-Related Gene Sets Show Significant Differences between Adjacent Cancer Samples and Tumor Samples

For BRCA, the mRNA expression profiles, together with matched clinical characteristics, were acquired with TCGA. We discovered four PyM-related gene sets on the GSEA website, which were called GO_PYRIMIDINE_CONTAINING_COMPOUND_CATABOLIC_PROCESS, GO_PYRIMIDINE_CONTAINING_COMPOUND_BIOSYNTHETIC_PROCESS, KEGG_PYRIMIDINE_METABOLISM, and GO_PYRIDINE_CONTAINING_COMPOUND_METABOLIC_PROCESS. First, we used GSEA to explore whether the genomes from the PyM-related gene sets show significant differences between the two groups of gene expression data. We found that only KEGG_PYRIMIDINE_METABOLISM gene set differs significantly between adjacent cancer samples and BRCA samples (normalized *p* value = 0.002 < 0.05) (Table 2, Figure 2(a)). Next, the core gene from the abovementioned gene set was screened, that is, the gene that has made the main contribution to the enrichment score of the gene set. We then selected 61 core genes for further analysis.

The Metascape Bioinformatics Tool was utilized for functional analysis of core genes to verify the above conclusion. The histogram and network diagram showed that the most enriched KEGG pathway was pyrimidine metabolism, suggesting that the core genes are indeed associated with PyM (Figure 2(b)).

### 3.2. Identification of PyM-Related Genes Associated with Prognosis in BRCA

According to the overall design and flow diagram of this study, we used the univariate Cox model to calculate the relationship between the expression levels of 61 selected PyM-related mRNAs and the patient's OS. It was found that there are 19 prognostic mRNAs in patients with BRCA. In total, 3 mRNAs (RRM2B, POLD2, and NME3) were selected upon multivariate Cox regression analysis to be the independent prognostic models (*p* < 0.05) (Table 3, Figure 3(a)). Afterwards, those chosen mRNAs were divided into risk (RRM2B and POLD2, hazard ratio: HR > 1) or protective (NME3, 0 < HR < 1) subtype.

Thereafter, alterations of those 3 screened mRNAs within BRCA were examined using cancer samples derived from the cBioPortal database. As a result, RRM2B had 16% cases of gene mutation, including gene amplification, missense mutation, and deep deletion; there were 5% of gene mutations in NME3, including gene amplification and deep deletion; 1.3% cases of POLD2 had gene mutation, including gene amplification and missense mutation (Figure 3(b)).

Expression levels of these 3 genes in BRCA and matched noncarcinoma tissues were differentially analyzed. As a result, the 3 genes in breast invasive cancer tissues were significantly upregulated (*p* < 0.05, Figure 3(c)).

### 3.3. Establishment and Confirmation of a Prognostic Signature

Then, the risk scores for all BRCA patients were determined according to the 3 prognostic mRNA expression as well as the regression coefficient (*β*) acquired through multivariate Cox regression. Risk score = (0.22065 × RRM2B level) + (−0.12697 × NME3 level) + (0.18280 × POLD2 level). The unique value of the risk score for each BRCA patient in the dataset can be calculated and was ranked in increasing order (Figure 4(a)). Thereafter, the median risk score was utilized to be the threshold for classifying 1108 BRCA cases as a high- or low-risk subgroups. As shown by KM curve analysis, high-risk patients had a dismal prognosis related to low-risk counterparts (*Log-rankp* < 0.001, Figure 4(c)). Figure 4(b) displays the risk score, OS (years) together with life status for 1108 cases from the dataset. As observed, a greater risk score indicated the worse survival status and shorter survival time of patients.

In addition, the chi-square test was adopted for revealing the association of risk score with clinical characteristics (Table 4), implying that a higher risk score was associated with T (tumor), N (node), and ER (estrogen receptor) status by IHC (immunohistochemistry) (*p* < 0.05).

### 3.4. The Three-mRNA Prognostic Signature Is Robust in BRCA Patients

The constructed 3-mRNA signature was used in the validation set including 1892 BRCA samples from the METABRIC database to validate its prediction ability. In the validation set, we used the same risk prediction model to calculate the risk score of each patient with BRCA and divided them into high-risk and low-risk subgroups using the median risk score. Conforming to prior results, high-risk patients showed markedly reduced survival time relative to low-risk patients in the validation set (Log-rank *p* value < 0.0001; Figure 5(c)). In addition, Figures 5(a) and 5(b) show the distribution of risk scores, life status, and survival time of 1892 BRCA patients. The above findings suggested that our constructed 3-mRNA signature contributed to the effective prediction of BRCA prognosis.

For verifying the superior effectiveness of the constructed 3-mRNA signatures on the single genes that make them up, we validated them through KM analysis. The results showed that when these 3 genes are used as an independent biomarker individually, the ability to predict the patient's survival is lower than the 3-mRNA signature (Log-rank *p* > 0.0007) (Figure 5(d)).

### 3.5. The Three-mRNA Signature Is an Independent Prognostic Indicator in BRCA Patients

For assessing the independence of our 3-mRNA signature-derived risk score from other clinical variables, we carried out univariate as well as multivariate Cox regression analysis. As shown in Figure 6(a), the distributions of diverse clinical factors in each subject were analyzed. First of all, upon univariate Cox regression, age, PR status, HER-2 status, ER status, M, N, stage, and risk score were significantly related to patients' survival with *p* values less than 0.05 (Figure 6(b)). Moreover, multivariate Cox regression analysis showed that the risk score generated from the 3-mRNA signature was an independent prognostic indicator, after adjusting for N (Figure 6(c)). And the risk score is the most robust parameter predicting the prognosis of patients with BRCA, because the probability of death in patients with high risk is 2.995 times that of patients with low risk.

In addition, a stratified analysis was carried out based on these clinical characteristics to determine the appropriate patient group for the risk prediction model. It turns out that the risk score is still remaining with the ability to predict OS within each subgroup of age, N, and HER-2 status (Figures 7(a), 7(b), and 7(d)). However, the risk score is more suitable for the subgroup of M0 (Figure 7(c)), which suggests that BRCA may be diseases that need further explanation.

## 4. Discussion

Breast cancer is one of the most common cancers among women, and susceptibility is explained by genetic, lifestyle, and environmental components [20]. BRCA is a major type of breast cancer; the main feature is that the tumor of this breast cancer infiltrates nearby tissues and has an obvious tendency to metastasize so far [21]. It is still a challenge to detect BRCA early. Therefore, creditable diagnostic approaches that attain high accuracy in prediction of the least genes should be developed to detect BRCA earlier [22]. Thanks to technological development, an increasing number of biomarkers are identified for the effective prediction of BRCA prognosis [23]. For instance, BRCA1 and BRCA2, the two primary BRCA suppressor genes, have been discovered in the 1990s [24]. Breast tumors carrying BRCA1 mutants are linked to basal-like and triple-negative phenotypes [25], but those with BRCA2 mutations are generally of the luminal subtype [26]. lncRNA OIP5-AS1 promotes breast cancer progression by regulating miR-216a-5p/GLO1 [27].CLIC2 is a useful biomarker for identifying breast cancer patients who could benefit from immune checkpoint blockade [28]. In addition, serum proteomics can be used in combination with bioinformatics analysis for the early detection of BRCA [29]. RS/DJ-1, the PTEN regulator [30], has been identified as the circulatory antigen discovered in serum samples of 37% new BRCA cases, rather than from normal subjects [31]. It can be seen that the methods for screening biomarkers are becoming increasingly diversified, and bioinformatics methods have gradually become a new attempt for us.

In recent years, the energy metabolism of tumors has become an indispensable research hotspot. Different from resting cells, tumor cells continuously supply deoxyribonucleoside triphosphates (dNTPs) resting in the de novo pathway, which thus facilitates the out-of-control tumor growth [1]. PyM represents a part of nucleotide metabolism to generate deoxy/ribonucleotides and nucleosides of pyrimidine bases (including uracil, thymine, and cytosine) [32]. Notably, the deoxyribonucleotide pool necessary for the proliferation of cells can be generated based on purine metabolism [33]. The persistent dNTP supply plays a crucial role in maintaining cancer cell survival [7]. Therefore, the permanent activation of the PyM gene from the beginning is necessary for growing tumors. KRAS drives tumor growth in pancreatic cancer by activating PyM [34]. Additionally, tumor cells are able to utilize diverse mechanisms for activating PyM genes and desensitizing the feedback regulatory pathway, thus resulting in allosteric suppression and maintaining the persistent cell nitrogen flow into the pathway producing dNTP along with ribonucleotide phosphate [35].

GSEA was performed in the present work for identifying gene sets associated with PyM to differentiate those clinical as well as molecular parameters for BRCA. In addition, the BRCA mRNA sequencing data along with the microarray data were acquired on TCGA database. Moreover, we applied the prognostic signature related to PyM (RRM2B, NME3, and POLD2) to predict OS for BRCA using Cox regression analysis. The as-constructed gene signature was adopted for classifying cases as high- or low-risk subgroups, identifying patients with BRCA with poor prognosis. Then, the METABRIC database was used to validate the signature prognosis prediction ability. Surprisingly, our prognostic model performed well on the KM analysis in 1892 BRCA patients. Stratification analysis indicated that the 3-mRNA signature-based risk score might independently predict the prognosis of each subgroup of age, N, and HER-2 status. However, the risk score is more suitable for the subgroup of M0 rather than M1, that is, the prognostic signature we selected is more suitable for BRCA that had not undergone distant metastasis, which suggests that our 3-mRNA signature may have great significance for the early diagnosis of BRCA. These findings suggested that our constructed 3-mRNA signature might serve as a biomarker for BRCA cases. Yet the low sample size was its limitation.

## 5. Conclusions

The present work first proposes the use of 3-mRNA signatures associated with PyM using bioinformatics methods for the prognosis of BRCA. In our study, cases who had high risk scores were found to show dismal prognostic outcome. The constructed 3-mRNA signature can be used as a prognostic marker for BRCA irrespective of additional clinicopathological factors. We believe that bioinformatics methods can be well combined with the early detection of breast cancer and can provide general guidance for the future application of molecular medicine combined biomarkers in other diseases. In the future, we will follow up with biological experiments and verify these biomarkers with our collaborators.

## Figures and Tables

**Figure 1:** The overall design and flow diagram.

**Figure 2:** Genes from the PyM-related gene sets show significant differences between adjacent cancer samples and tumor samples. (a) Enrichment plots of 4 gene sets. (b, c) Functional enrichment analysis. (The figure is colored by the degree of enrichment. The darker the color, the greater the number of genes enriched in this type of pathway or biological process).

**Figure 3:** Identification of PyM-related genes associated with prognosis in BRCA. (a) The coefficients of the 3 genes, red for risk factors and blue for protective factor. (b) Selected genes' alteration with the study. (c) Different expression of 3 selected genes (^∗^*p* < 0.05, ^∗∗^*p* < 0.01, ^∗∗∗^*p* < 0.001, and ^∗∗∗∗^*p* < 0.0001).

**Figure 4:** Establishment and confirmation of a prognostic signature. (a) mRNA risk score distribution in each patient. (b) Survival time and status of patients in order of the value of risk scores. (c) The risk score calculated from three-mRNA signature predicts overall survival in the patients with BRCA.

**Figure 5:** The three-mRNA prognostic signature is robust in BRCA patients. (a–c) Validation of prognostic efficiency for three-mRNA signature within 1892 BRCA patients from the METABRIC database. (d) Performance of 3 genes when they are used as a single biomarker.

**Figure 6:** The risk score generated from the 3-mRNA signature as a prognostic indicator is independent from other clinical variables. (a) Distribution of the clinicopathological parameters in BRCA patients with low-risk score to high-risk score. (b) Univariate Cox regression analysis of OS. (c) Multivariate Cox regression analysis of OS.

**Figure 7:** Stratified analysis: (a) age; (b) Her-2 status by IHC; (c) M classification (M0: no distant metastasis; M1: distant metastasis); (d) N classification (N0: no lymph node metastasis; N1: 1–3 lymph node metastasis; N2: 4–9 lymph node metastasis; N3: ≥10 lymph node metastasis).

**Table 1:** Clinical parameters of patients with BRCA from TCGA.

Clinical parameters	*n*	%	Dead number
Age (years)			
≥58	581	52.44	89
<58	527	47.56	66
pTNM stage			
Stage I	183	16.52	16
Stage II	626	56.50	69
Stage III	251	22.65	44
Stage IV	20	1.80	15
Unknown	28	2.53	11
Primary tumor			
T1	282	25.45	33
T2	641	57.85	81
T3	138	12.45	25
T4	40	3.61	15
Unknown	7	0.63	1
Regional lymph nodes			
N0	553	49.91	48
N1	332	29.96	59
N2	120	10.83	22
N3	79	7.13	15
Unknown	24	2.17	11
Metastasis			
M0	918	82.85	124
M1	22	1.99	17
Unknown	168	15.16	14
Person neoplasm status			
With tumor	96	8.67	88
Tumor-free	882	79.60	39
Unknown	130	11.73	15
ER status by IHC			
Negative	239	21.57	42
Positive	814	73.47	102
Unknown	55	4.96	11
PR status by IHC			
Negative	345	31.14	57
Positive	705	63.63	88
Unknown	58	5.23	10
HER-2 status by IHC			
Negative	567	51.17	59
Positive	164	14.80	23
Unknown	377	34.03	73

**Table 2:** Gene sets enriched in patients with BRCA and their core genes (1108 samples).

GS follow link to MSigDB	Size	NOM *p* value	FDR *q* value	Core gene list	Core enrichment
KEGG_PYRIMIDINE_METABOLISM	61	0.002	0.013	POLD3, NUDT2, POLR3A, RRM2B, TXNRD1, DUT, UPRT, UCK2, POLR1B, POLR2L, POLA1, NT5C, TXNRD2, NME, NME6, PNPT1, UMPS, POLR1C, NME2, NT5C3A, POLR3C, CAD, UCKL1, CMPK2, POLR2D,NME1-NME2, POLR1A, NT5M, ENTPD8, DCK, POLE3, CTPS2, PRIM1,ZNRD1, RRM1, ENTPD6, POLR2I, PRIM2, POLR2K, POLE, PNP,POLR2G, POLD4, POLD1, POLD2, NME3, CTPS1, NME1, ITPA, POLR2J,TYMS, CANT1, NME4, POLA2, TYMP, TK1, POLE2, POLR2H, DTYMK,RRM2, POLR3K	Yes
GO_PYRIMIDINE_CONTAINING_COMPOUND_CATABOLIC_PROCESS	15	0.127	0.127	DUT, APOBEC3A, NT5C, APOBEC3H, NT5C3A, TDG, MBD4, NT5M,UNG, TET3, APOBEC3B, SMUG1, NTHL1, TYMP, DCTPP1	Yes
GO_PYRIMIDINE_CONTAINING_COMPOUND_BIOSYNTHETIC_PROCESS	26	0.12	0.12	DUT, UPRT, UCK2, GPAT4, NME2P1, NME7, PRPS1, NME6, UMPS,NME2, CAD, AGPAT3, UCKL1, CMPK2, DCK, CTPS2, LCLAT1, CDS1,NME3, CTPS1, NME1, TYMS, NME4, TYMP, TK1, DTYMK	Yes
GO_PYRIDINE_CONTAINING_COMPOUND_METABOLIC_PROCESS	15	0.333	0.333	PSAT1, IDO1, SLC5A8, ACMSD, NUDT17, PNPO, NADSYN1, KMO,NAPRT, QPRT, PDXP, IDH2, PARP9, PNP, PARP10	Yes

**Table 3:** Information of the 3 filtered mRNAs.

mRNA	Ensemble ID	*β* (Cox)	HR	*p*
RRM2B	**ENSG00000048392**	**0.22065**	**1.24688**	**0.0088**
NME3	**ENSG00000103024**	**-0.12697**	**0.88076**	**0.0104**
POLD2	**ENSG00000106628**	**0.18280**	**1.20058**	**0.0138**

**Table 4:** The relation between risk score and clinical features.

Clinical feature	Risk score		*X* ^2^	*p*
	High risk *n* (%)	Low risk *n* (%)		
Age			0.044	0.835
≥58	285 (26.27)	280 (25.81)		
<58	259 (23.87)	261 (24.05)		
T			8.930	**0.030**
T1	126 (11.65)	153 (14.14)		
T2	333 (30.78)	294 (27.17)		
T3	59 (5.45)	78 (7.21)		
T4	23 (2.13)	16 (1.47)		
N			10.250	**0.017**
N0	250 (23.47)	296 (27.79)		
N1	171 (16.06)	152 (14.27)		
N2	72 (6.76)	47 (4.41)		
N3	38 (3.57)	39 (3.67)		
M			0.003	0.960
M0	478 (51.73)	425 (46.00)		
M1	11 (1.19)	10 (1.08)		
Stage			5.344	0.148
I	77 (7.25)	104 (9.79)		
II	309 (29.10)	307 (28.91)		
III	132 (12.43)	114 (10.73)		
IV	9 (0.85)	10 (0.94)		
Person neoplasm cancer status			3.477	0.062
Tumor-free	420 (43.66)	448 (48.38)		
With tumor	55 (5.94)	39 (2.02)		
PR status by IHC			3.266	0.071
Negative	184 (17.83)	158 (15.31)		
Positive	330 (31.98)	360 (34.88)		
ER status by IHC			8.363	**0.004**
Negative	138 (13.33)	100 (9.66)		
Positive	377 (36.43)	420 (59.90)		
HER-2 status by IHC			1.049	0.306
Negative	283 (39.42)	274 (38.16)		
Positive	86 (11.98)	75 (10.44)		

## Data Availability

The datasets generated and analyzed during the current study are available in TCGA (http://cancergenome.nih.gov/) and METABRIC (https://ega-archive.org/dacs/EGAC00001000484) database.

## Abbreviations

BRCA: Breast invasive carcinoma
PyM: Pyrimidine metabolism
TCGA: The Cancer Genome Atlas
GSEA: Gene set enrichment analysis
KM: Kaplan-Meier
METABRIC: Molecular Taxonomy of Breast Cancer International Consortium
OS: Overall survival
IHC: Immunohistochemistry.
